The article "Effect of Electromyographic Biofeedback Therapy on Muscle Strength Recovery in Children with Guillain–Barré Syndrome" was published in 2021. Journal: J Healthc Eng.

# Effect of Electromyographic Biofeedback Therapy on Muscle Strength Recovery in Children with Guillain–Barré Syndrome

**DOI:** 10.1155/2021/1220368

**Published:** 2021-12-23

**Authors:** Qianqian Liu, Jianhua Xue, Pingping Zhao, Yue Ling, Suzhe Liu, Yakun Du, Ning Han, Mingxia Liu, Wei Di

**Affiliations:** ^1^Department of Neurological Rehabilitation, Hebei Children's Hospital, Shijiazhuang 050031, Hebei, China; ^2^Department of Neurology Shijiazhuang the Third Hospital, Hebei Children's Hospital, Shijiazhuang 050031, Hebei, China; ^3^Quality Control Department, Hebei Children's Hospital, Shijiazhuang 050031, Hebei, China; ^4^Department of Neurology, Hebei Children's Hospital, Shijiazhuang 050031, Hebei, China; ^5^Hyperbaric Oxygen Department, Hebei Children's Hospital, Shijiazhuang 050031, Hebei, China

## Abstract

GBS, as an immune-mediated acute inflammatory peripheral neuropathy (Tan and Halpin et al.), with the characteristics of acute onset and rapid progression, is mainly manifested with damages in nerve root and peripheral nerve. The purpose of the study was to investigate the effect of electromyographic biofeedback therapy on muscle strength recovery in children with Guillain–Barré syndrome (GBS). A total of 62 GBS children patients admitted to our hospital from June 2014 to December 2018 were selected and divided into control group (*n* = 30) and experimental group (*n* = 32) according to the order of admission. The children patients in the control group received physical therapy combined with occupational therapy (PT + OT), while based on the treatment in the control group, the experimental group children patients were treated with electromyographic biofeedback therapy. After that, the recovery of nerve and muscle at different time points, muscle strength score, gross motor function measure (GMFM) score, and Barthel index (BI) score of the children patients before and after treatment were compared between the two groups. There were no significant differences in the recovery of nerve and muscle of the children patients between the two groups at *T*_0_ and *T*_1_ (*P* > 0.05), and the recovery of nerve and muscle of the children patients in the experimental group was significantly better than that in the control group at *T*_2_, *T*_3_, and *T*_4_ (*P* < 0.001); the muscle strength score, GMFM score, and BI score of the children patients in the experimental group were significantly better than those in the control group after treatment (*P* < 0.001). The application of electromyographic biofeedback therapy for the treatment of GBS can effectively relieve clinical symptoms, promote rapid recovery, and improve treatment efficacy in children patients, which is worthy of application and promotion.

The article "Effect of Electromyographic Biofeedback Therapy on Muscle Strength Recovery in Children with Guillain–Barré Syndrome" was published in 2021. Journal: J Healthc Eng.

## 1. Introduction

The [1, 2] common clinical symptom of GBS is ascending paralysis which results in symmetrical leg weakness in patients. In addition, the GBS patients typically suffer from the weakness of extremities, body, and even cranial nerve in just a few hours and several days [3–5], and their lower limbs are more affected than upper limbs, which finally leads to flaccid paralysis and the weakness or disappearance of tendon reflex. Generally, in the early stage of GBS, the disappearance of tendon reflex, dysfunction, and even speech disorders such as aphasia may occur in children patients, and some children have mild muscle atrophy or disuse atrophy after long-term staying in bed [6–9]. GBS can affect all ages, with the annual incidence of 0.6∼1.9 per 100,000 persons, which is slightly higher in men than in women. At present, the clinical treatment measures taken for GBS are enhanced respiratory management, anti-infective therapy, nutrition support, and rehabilitation training, which can improve body dysfunction, but these are still far away from the desired effect [10–12]. With the advancement of medical rehabilitation technology, early rehabilitation is critical to GBS treatment, and the electromyographic biofeedback therapy, which has been widely applied in preventive medicine, clinical medicine, and rehabilitation medicine since the 80s, has contributed positively to the recovery of muscle and nerve [13–15]. Clinical studies have found that electromyographic biofeedback therapy can promote rapid recovery in children and achieve a significant clinical effect. In order to further investigate the effect of electromyographic biofeedback therapy on muscle strength recovery in GBS children, a total of 62 GBS children patients admitted to our hospital from June 2014 to December 2018 were selected as the study subjects. The studies are summarized and reported as follows.

## 2. Materials and Methods

### 2.1. General Information

A total of 62 GBS children patients admitted to our hospital from June 2014 to December 2018 were selected and divided into control group (*n* = 30) and experimental group (*n* = 32) according to the order of admission.

### 2.2. Inclusion Criteria

(1) Children patients met the diagnostic criteria for acute and chronic GBS made by Asbury and the American Academy of Neurology. (2) Children patients had stable conditions and had no respiratory failure. (3) Children patients had no tumors after brain MRI or CT examination and had no progressive brain diseases or other neurodegenerative diseases. (4) Children patients and their family members had good compliance. (5) Children patients had complete clinical data. (6) This study was approved by the Hospital Ethics Committee, and the children patients' family members were informed of the purpose and process of this study and signed the informed consent.

The article "Effect of Electromyographic Biofeedback Therapy on Muscle Strength Recovery in Children with Guillain–Barré Syndrome" was published in 2021. Journal: J Healthc Eng.

### 2.3. Exclusion Criteria

(1) Children patients had diseases in heart, liver, kidneys, blood system, and others. (2) Children patients had epilepsy. (3) Children patients had no skin damage, fracture, and metal implant in treatment sites.

### 2.4. Methods

The children patients in the control group were treated with PT + OT, and the specific measures were as follows. (1) Medical staff should closely monitor all vital signs of the children patients and regularly help them turn over to discharge respiratory secretions and ensure smooth breathing. For the children patients suffering from dysphagia and coughing when drinking, nutrition supports by nasal feeding should be given to ensure that the daily intake of vitamins and calories meets the standards required for human body. At the same time, clinical symptoms such as corneal ulcer, pneumonia, and atelectasis should be prevented, and if children patients had cardiac arrhythmia, blood pressure changes, and constipation, they should be given symptomatic treatment. (2) The children patients should receive an intravenous injection of 5% glucose injection (manufacturer: Anhui Guosen Pharmaceutical Co., Ltd.; State Food and Drug Administration approval number: H34021537; specification: 250 ml: 25g), and on basis of that, they should also be given an intramuscular injection of 0.2 g of vitamin B_6_ injection (manufacturer: Shandong Yijian Pharmaceutical Co., Ltd.; State Food and Drug Administration approval number: H20058778; specification: 2 ml: 0.1 g) once a day. Besides, intramuscular injection of 0.5 mg of vitamin B_12_ (manufacturer: Jiangsu Hengfeng Pharmaceutical Co., Ltd.; State Food and Drug Administration approval number: H32020230; specification: 1 ml: 0.5 mg) should be performed once daily, and the intravenous injection of 0.4 g/kg of *γ*-globulin (manufacturer: Shanxi Kangbao Biological Products Co., Ltd.; State Food and Drug Administration approval number: S19994004; specification: 5%, 50 ml/vial, or 2.5 g/vial) was also conducted once a week for one month. (3) Medical staff should firstly ask the children patients and their family members to move limb joints on their own to ensure that joint activity levels are within a reasonable range. Secondly, physical therapists should develop a reasonable rehabilitation program based on the actual conditions of the children patients, implement specific training on children patients' coordination, balance, and endurance and intervene in their dietary habits. Finally, the children patients should be guided to conduct step training and hand exercises from simple to complex, so as to help them gradually adapt to this type of rehabilitation.

The article "Effect of Electromyographic Biofeedback Therapy on Muscle Strength Recovery in Children with Guillain–Barré Syndrome" was published in 2021. Journal: J Healthc Eng.

Based on the treatment in the control group, the children patients in the experimental group were given electromyographic biofeedback therapy, and the specific measures were as follows. The children in the experimental group were treated by myoelectric biofeedback therapy apparatus (manufacturer: Shanghai Nuocheng Electric Co., Ltd.; Shanghai Food and Drug Administration certified number: (2010) 2211141; model: MyoNet-COW type). After the children patients took sitting positions, fixed electrodes were placed on 4 cm above lateral malleus and the muscle belly of tibialis anterior muscle, and meanwhile, the reference electrodes were placed on knee joints, with semiactive mode. The output intensity of electrical stimulation was adjusted manually before treatment and 75% of the mean value of surface myoelectricity during the first three tibialis anterior muscle contractions was used as the trigger threshold. When the apparatus started, the children patients should be instructed to contract their tibialis anterior muscles, and the occurrence of triggering electrical stimulation represented that the threshold was triggered. Then, medical staff should help the children patients to finish foot dorsiflexion, with the apparatus frequency of 60 Hz and the intensity of 25 mA (which could be adjusted properly), and the movement lasted for 8 s at a time, with the interval of 15 s; the number of feedback was 35 times, 25 min/time, 6 times a week. The children patients in both groups were treated continuously for 3 months.

### 2.5. Observation Indexes

The recovery of nerve and muscle was evaluated by the nervous system assessment scale and muscle recovery assessment scale both made by our department, with each scale scoring 20 points in total, and lower scores represented better recovery of nerve and muscle. Before treatment, 2 weeks, 1 month, 3 months, and 6 months were set as *T*_0_, *T*_1_, *T*_2_, *T*_3_, and *T*_4_, respectively, and the recovery of nerve and muscle at different time points was compared between the two groups.

Muscle strength and limb mobility of the children patients were evaluated by the Lovett manual muscle test, with the total score of 5 points, whose higher scores indicated better muscle strength, and the GMFM scale, scoring 3 points in total, whose higher scores represented better limb mobility.

The daily living ability of the children patients was assessed by the BI scale, with a total score of 100 points, and higher scores represented better daily living ability.

The article "Effect of Electromyographic Biofeedback Therapy on Muscle Strength Recovery in Children with Guillain–Barré Syndrome" was published in 2021. Journal: J Healthc Eng.

### 2.6. Statistical Treatment

The selected data processing software for this study was SPSS20.0, and GraphPad Prism 7 (GraphPad Software, San Diego, USA) was used to draw the pictures of the data. Measurement data were tested by *t*-test, and enumeration data were tested by *X*^2^ test and normality test. The differences had statistical significance when *P* < 0.05.

## 3. Results

### 3.1. Comparison of General Information of the Children Patients between the Two Groups

There were no significant differences in gender, age, BMI, pathological type, and place of residence between the two groups, with comparability (*P* > 0.05), as detailed in Table 1.

### 3.2. Comparison of Nerve Recovery of the Children Patients between the Two Groups before and after Treatment

There were no significant differences between the two groups in nerve recovery at *T*_0_ and *T*_1_ (*P* > 0.05), and the nerve recovery in the experimental group at *T*_2_, *T*_3_, and *T*_4_ were significantly better than that in the control group (*P* < 0.05), as shown in Table 2.

### 3.3. Comparison of Muscle Recovery of the Children Patients between the Two Groups before and after Treatment

There were no significant differences in muscle recovery between the two groups at *T*_0_ and *T*_1_ (*P* > 0.05), and the muscle recovery in the experimental group at *T*_2_, *T*_3_, and *T*_4_ was significantly better than that in the control group (*P* < 0.05), as detailed in Figure 1.

### 3.4. Comparison of Muscle Strength Score between the Two Groups

The muscle strength in the experimental group after treatment was significantly better than that in the control group (*P* < 0.05), as detailed in Figure 2.

### 3.5. Comparison of GMFM Score between the Two Groups

The GMFM score in the experimental group after treatment was significantly better than that in the control group (*P* < 0.05), as detailed in Figure 3.

### 3.6. Comparison of BI Score between the Two Groups

The BI score in the experimental group after treatment was significantly better than that in the control group (*P* < 0.05), as detailed in Figure 4.

## 4. Discussion

The case fatality rate of GBS is about 5%; however, after treatment and rehabilitation, the neurological function of 50% of children patients basically recovers within weeks to months, about 20%∼30% requires assisted ventilation, and only 10%∼15% suffers from persistent neurological dysfunction [16–18]. With the advancement of medical rehabilitation technology, early rehabilitation is critical to GBS treatment, and the electromyographic biofeedback therapy, which has been widely applied in preventive medicine, clinical medicine, and rehabilitation medicine since the 80s, has contributed positively to the recovery of muscle and nerve [13–15]. Combined with GBS patients' conditions, electromyographic biofeedback can take staged treatment measures according to different stages of the disease, including muscle excitability feedback training, muscle endurance training, coordination function training, and muscle relaxation feedback training, so as to improve or restore the stimulated muscles or muscle groups. Children patients usually have poor compliance and low treatment cooperation, which causes poor therapeutic effect; electromyographic biofeedback can provide feedback animation windows through audio-visual pathways to improve the cooperation and compliance of the children patients to the treatment, and thus the children patients can actively participate in the rehabilitation and promote their rapid recovery [19–22]. Biofeedback therapy is one of the clinically important treatment measures, mainly used for the rehabilitation of neuromuscular and injurious diseases, such as GBS, spinal cord injury, facial palsy, peripheral nerve injury, cerebral infarction in children, child cerebral palsy, sweeny, and bone stiffness. In recent years, with the development of electromyographic biofeedback therapy, its application has been increasingly expanding. This study showed that the GMFM score in the experimental group was significantly better than that in the control group after treatment (*P* < 0.001), which is in line with the findings of Siddiqui et al. [23], who have stated that the GMFM score in the treatment group is higher than that in the control group (*P* < 0.05), with statistically significant differences, indicating that the implementation of electromyographic biofeedback therapy in GBS children can effectively improve limb mobility and promote rapid physical rehabilitation. The application of electromyographic biofeedback therapy for the treatment of GBS can effectively relieve clinical symptoms, promote rapid recovery, and improve treatment efficacy in children patients, which is worthy of application and promotion.

The article "Effect of Electromyographic Biofeedback Therapy on Muscle Strength Recovery in Children with Guillain–Barré Syndrome" was published in 2021. Journal: J Healthc Eng.

## 5. Conclusion

In conclusion, electromyographic biofeedback therapy, with obvious effect on the rehabilitation of GBS, can shorten treatment time, promote rapid recovery, and provide reliable and precise rehabilitation support for GBS children to obtain higher quality of life or return to society, which is worthy of application and promotion.

## Figures and Tables

**Figure 1:** Comparison of muscle recovery of the children patients between the two groups before and after treatment ($\bar{x}\pm s$). Note: the abscissa represented the *T*_0_, *T*_1_, *T*_2_, *T*_3_, and *T*_4_, respectively, while the ordinate represented muscle recovery, points. In the experimental group, the muscle recovery scores at *T*_0_, *T*_1_, *T*_2_, *T*_3_, and *T*_4_ were 18.12 ± 1.76 points, 15.03 ± 2.2 points, 9.32 ± 0.66 points, 4.36 ± 0.52 points, and 1.5 ± 0.25 points, respectively. In the control group, the muscle recovery scores at *T*_0_, *T*_1_, *T*_2_, *T*_3_, and *T*_4_ were 18.03 ± 1.96 points, 15.08 ± 2.03 points, 12.11 ± 1.41 points, 7.32 ± 1.19 points, and 3.88 ± 0.39 points, respectively. ^*∗*^ indicated that there were no significant differences in muscle recovery at *T*_2_ between the two groups (*t* = 10.081, *P* ≤ 0.01). ^*∗∗*^ indicated that there were no significant differences in muscle recovery at *T*_3_ between the two groups (*t* = 12.830, *P* ≤ 0.01). ^*∗∗∗*^ indicated that there were no significant differences in muscle recovery at *T*_4_ between the two groups (*t* = 28.791, *P* ≤ 0.01).

**Figure 2:** Comparison of muscle strength score between the two groups ($\bar{x}\pm s$). Note: the abscissa represented before and after treatment, while the ordinate represented muscle strength score, points. In the experimental group, the muscle strength scores before and after treatment were 0.53 ± 0.35 points and 4.21 ± 0.77 points, respectively. In the control group, the muscle strength scores before and after treatment were 0.49 ± 0.91 points and 3.12 ± 0.89 points, respectively. ^*∗*^ indicated that there were significant differences in muscle strength scores in the experimental group before and after treatment (*t* = 24.612, *P* ≤ 0.01). ^*∗∗*^ indicated that there were significant differences in muscle strength scores in the control group before and after treatment (*t* = 11.317, *P* ≤ 0.01). ^*∗∗∗*^ indicated that there were significant differences in muscle strength scores after treatment between the two groups (*t* = 5.166, *P* ≤ 0.01).

**Figure 3:** Comparison of the GMFM score between the two groups ($\bar{x}\pm s$). Note: the abscissa represented before and after treatment, while the ordinate represented GMFM score, points. In the experimental group, the GMFM scores before and after treatment were 0.35 ± 0.86 points and 2.21 ± 0.68 points, respectively. In the control group, the GMFM scores before and after treatment were 0.41 ± 0.78 points and 1.53 ± 0.48 points, respectively. ^*∗*^ indicated that there were significant differences in GMFM scores in the experimental group before and after treatment (*t* = 9.597, *P* ≤ 0.01). ^*∗∗*^ indicated that there were significant differences in GMFM scores in the control group before and after treatment (*t* = 6.698, *P* ≤ 0.01). ^*∗∗∗*^ indicated that there were significant differences in GMFM scores after treatment between the two groups (*t* = 4.521, *P* ≤ 0.01).

The article "Effect of Electromyographic Biofeedback Therapy on Muscle Strength Recovery in Children with Guillain–Barré Syndrome" was published in 2021. Journal: J Healthc Eng.

**Figure 4:** Comparison of BI score between the two groups. Note: the abscissa represented before and after treatment, while the ordinate represented BI score, points. The BI scores in the experimental group before and after treatment were 61.23 ± 6.33 points and 89.12 ± 10.15 points, respectively. The BI scores in the control group before and after treatment were 60.88 ± 5.37 points and 77.77 ± 9.89 points, respectively. ^*∗*^ indicated that there were significant differences in BI scores in the experimental group before and after treatment (*t* = 13.189, *P* ≤ 0.01). ^*∗∗*^ indicated that there were significant differences in BI scores in the control group before and after treatment (*t* = 8.220, *P* ≤ 0.01). ^*∗∗∗*^ indicated that there were significant differences in BI scores between the two groups after treatment (*t* = 4.454, *P* ≤ 0.01).

**Table 1:** Comparison of general information of the children patients between the two groups (*n* (%)).

	Experimental group (*n* = 32)	Control group (*n* = 30)	*X* ^2^ or *t*	*P*
Gender			0.001	0.974
Male	18 (56.25)	17 (56.67)		
Female	14 (43.75)	13 (43.33)		
Age (years old)	9.27 ± 1.3	9.31 ± 1.1	0.130	0.896
BMI (kg/m^2^)	17.55 ± 3.42	17.49 ± 3.31	0.070	0.944
Pathological type				
AIDP	10 (31.25)	9 (30.00)	0.011	0.915
AMAN	8 (25.00)	7 (23.33)	0.023	0.878
AMSAN	9 (28.13)	7 (23.33)	0.185	0.667
MFS	5 (15.63)	7 (23.33)	0.589	0.443
Place of residence			0.242	0.622
Urban area	18 (56.25)	15 (50.00)		
Rural area	14 (43.75)	15 (50.00)		

**Table 2:** Comparison of nerve recovery of the children patients between the two groups before and after treatment ($\bar{x}\pm s$).

Group	*n*	*T*_0_	*T*_1_	*T*_2_	*T*_3_	*T*_4_
Experimental group	32	17.33 ± 2.55	13.57 ± 1.38	9.22 ± 1.54	5.11 ± 0.98	2.12 ± 0.53
Control group	30	17.41 ± 2.47	14.11 ± 1.56	12.35 ± 1.61	7.86 ± 1.23	5.21 ± 0.88
*t*		0.125	1.445	7.823	9.767	16.870
*P*		0.900	0.153	<0.001	<0.001	<0.001

## Data Availability

The datasets used and/or analyzed during the current study are available from the corresponding author on reasonable request.
